This article has been retracted.

# Neurogenic Stunned Myocardium: A Literature Review

**DOI:** 10.7759/cureus.3129

**Published:** 2018-08-10

**Authors:** Asad Ali, Malik Qistas Ahmad, Muhammad Bilal Malik, Zara Z Alvi, Waleed Iftikhar, Deepak Kumar, Usama Nasir, Nouman Safdar Ali, Zohaib Sayyed, Risham Javaid, Neha Waqas, Shahzad Ahmed Sami, Abbas M Cheema

**Affiliations:** 1 Medicine, CMH Lahore Medical College and Institute of Dentistry, Lahore, PAK; 2 Hematology-Oncology, University of Arizona Cancer Center, Tucson, USA; 3 Internal Medicine, Shifa College of Medicine, Islamabad, PAK; 4 Internal Medicine, CMH, Lahore Medical College, Lahore, PAK; 5 Internal Medicine, CMH Lahore Medical College and Institute of Dentistry, Lahore, PAK; 6 Internal Medicine, Jinnah Postgraduate Medical Centre, Karachi, PAK; 7 Medicine, Jinnah Hospital/Allama Iqbal Medical College, Lahore, PAK; 8 Pediatrics, Shaikh Khalifa Bin Zayed Al-Nahyan Medical and Dental College, Bahawalpur, PAK; 9 Medicine, Akhter Saeed Trust Hospital, Lahore, PAK; 10 Surgery, Shaikh Khalifa Bin Zayed Al Nahyan Medical & Dental College, Broken Bow, PAK; 11 Internal Medicine, CMH Medical and Dental College, Lahore, PAK; 12 Internal Medicine, Combined Military Hospital, Lahore, PAK

**Keywords:** coronary heart disease, acute coronary syndrome, troponin, stroke, electrocardiogram, autonomic nervous system, left ventricular dysfunction, cardiomyopathy, neurogenic

## Abstract

Neurogenic stunned myocardium (NSM) is defined as the occurrence of cardiac abnormalities due to neurological events such as stroke, seizures, etc. These events lead to dysfunction of the autonomic nervous system (ANS) and ultimately cause injury to the myocardium. The clinical features seen in NSM include elevated troponin level, left ventricular dysfunction, and changes on the electrocardiogram (ECG). However, these features are also seen in Takotsubo cardiomyopathy as well as in an acute coronary syndrome (ACS). Hence, diagnosing the condition by clinical presentation alone is difficult. Thus, a patient of NSM who is at increased risk of developing coronary heart disease may require invasive procedures such as cardiac catheterization to rule out ACS. This review aims at raising awareness about NSM among physicians so that management of patients can be individualized.

## Introduction and background

Annually, approximately 800,000 people in the US suffer from stroke, including recurrences. A person has a stroke in the country roughly every 40 seconds, and there is a stroke-related death every four minutes [1]. Stroke is also a major cause of functional disability [2]. Moreover, acute stroke often leads to cardiac complications [3]. These include arrhythmias, ventricular dysfunction, myocardial ischemia or infarction, as well as sudden cardiac death [4]. Chin et al. showed that in about 13% of patients who suffered a cerebrovascular incident, there was an associated myocardial infarction (MI) seen within three days [5]. Statistics show that the most common non-neurological causes of death seen in the first month of a cerebrovascular stroke were related to the cardiovascular system [6]. Moreover, cardiac events are also the leading cause of mortality during the long-term follow-up of patients with cerebrovascular stroke [7]. The risk of a myocardial infarction (MI) can be as high as 2% even a few years after a stroke [8].

Neurogenic stunned myocardium (NSM) is defined as the occurrence of cardiac abnormalities due to neurological events such as stroke, seizures, etc. These events lead to the dysfunction of the autonomic nervous system and ultimately can lead to several different types of cardiac disorders [9-10]. Like MI, NSM can cause electrocardiogram (ECG) changes suggestive of ischemia, cardiac dysfunction, raised troponin levels, and regional wall motion abnormalities. The mechanism considered responsible for NSM is the increase in catecholamine levels due to brain damage occurring from autonomic dysfunction. Despite having a similar presentation, NSM differs from myocardial infarction as there is no significant coronary vessel block seen in this condition.

Like myocardial infarction, another condition with a presentation similar to NSM is Takotsubo cardiomyopathy. Both NSM and Takotsubo cardiomyopathy have similar pathophysiology and presentations. However, wall motion abnormality is a difference noted between the two. NSM is usually associated with global hypokinesis, whereas Takotsubo cardiomyopathy leads to regional wall motion abnormalities. Due to these similarities, some physicians consider them as a single condition falling under the category of stress-induced cardiomyopathy.

It is challenging to differentiate between NSM and acute MI. Bulsara et al. have devised certain guidelines to help discriminate between these two similar entities in patients with subarachnoid hemorrhage. NSM can be distinguished from acute MI by the following: (1) lack of pre-existing heart disease; (2) cardiac dysfunction of recent onset with ejection fraction < 40%; (3) wall motion abnormalities which do match ECG changes; (4) low troponin levels, i.e., less than 2.8 ng/ml in patients with a low ejection fraction [11]. However, it should be noted that these guidelines do not apply to patients with ischemic strokes as they are likely to have concomitant heart disease.

## Review

Pathophysiology

It has been shown that autonomic dysfunction and adverse cardiac events after a stroke are associated with the involvement of the insular cortex of the brain. This area connects with other areas of the brain including the limbic system and helps in integrating the autonomic, motor, and sensory functions. In NSM, the insular cortex plays a key role in balancing the sympathetic and parasympathetic nervous systems.

The limbic and autonomic regulatory control of the cardiovascular system is carried out by the insula, with the help of baroreceptors in the insular cortex that helps alter the blood pressure and heart rate. Any stimulation of the insula results in an alteration of these parameters. Moreover, any lesions involving the insular cortex in the brain cause an increased release of norepinephrine leading to left ventricular dysfunction. The effects seen due to the stimulation of right or left insula are different. Right insular stimulation results in sympathetic effects such as an increase in the heart rate (tachycardia) and an increase in blood pressure (hypertension). In comparison, the stimulation of the left insula results in parasympathetic effects, such as bradycardia and a reduction in blood pressure. Conversely, a stroke involving the right insular region will cause lowered sympathetic regulation and an increase in parasympathetic effects [7]. The reverse will be seen in left insular stroke. A stroke involving bilateral insular regions may lead to a decrease in heart rate variability. It is important to note that the involvement of the insular cortex on either side is associated with an increase in cardiovascular morbidity and mortality. As far as the parietal lobe is concerned, its role in NSM is ambiguous. More extensive research needs to be done before establishing its importance.

The principal mechanism of NSM is an increased sympathetic stimulation. The initiating event is an influx of catecholamines because of a lesion in the brain or due to excessive stress. Eventually, cardiac injury occurs which can be in the form of (a) ischemic insult due to inability to meet the increased myocardial demand [9]; (b) direct myocardial toxicity due to the increased levels of catecholamines; and/or (c) vasospasm of the coronary vessels in response to the increased catecholamines. The direct toxicity of the catecholamines occurs due to an increased calcium influx in the cardiac muscle cells. This occurs because the beta-adrenergic receptors are stimulated by increased catecholamines, which in turn lead to the opening of calcium channels. The increased calcium influx in cardiomyocytes leads to contractile dysfunction and lowering of adenosine triphosphate (ATP), ultimately leading to cell death.

The histological changes seen in NSM include transient myofibrillar degeneration, also known as myocytolysis. Myocytolysis is characterized by multiple foci of subendocardial hemorrhage seen around the epicardial nerves and is indicative of actual myocardial stress. As the myocytolysis affects the subendocardial region which is also the site of the cardiac conducting system, arrhythmias are seen frequently in NSM.

Troponin levels

Stroke patients can develop NSM which might remain asymptomatic and thus be missed. An increase in troponin levels might represent the only sign of cardiac damage in such patients and can be seen without chest pain and abnormalities on the ECG or the echocardiogram. Faiz et al. showed that approximately 53% of patients with acute ischemic stroke had raised troponin levels [12]. However, only 6% of these met the diagnostic criteria for myocardial infarction. Jensen and his colleagues showed that troponin levels were found increased in only 3% of patients without obvious coronary heart disease [13].

Raised troponin levels can also be indicative of a poor prognosis in stroke patients. According to Ghali et al., in patients of ischemic stroke, troponin showed a sensitivity of 0.27, specificity of 0.94, and a likelihood ratio of 4.5 when it was used to predict a poor outcome. Moreover, troponin levels also showed a correlation between the severity of stroke [14]. Jensen et al. also showed that elevated troponin levels correlated with increased risk of early death as well as an increased two-year mortality. Despite these findings, the National Institutes of Health Stroke Scale (NIHSS) has been found to be a superior prognostic predictor than troponin, with a higher sensitivity (0.78), specificity (0.96), and likelihood ratio (17.7). Despite there being several studies evaluating troponin levels in patients with acute ischemic stroke, these are not uniform and vary in terms of laboratory assay, laboratory references, and cut-offs.

Electrocardiographic features

Approximately 60%-90% of patients with cerebral infarction also demonstrate abnormal ECG findings, the most common of which is a prolonged QT interval. The second most common abnormal ECG finding in patients with cerebral infarctions is a T-wave inversion, followed by ST-segment depression. Atrial fibrillation is the most common abnormal rhythm seen in these patients, followed by sinus tachycardia. Approximately 8% of patients with cerebral infarction showed a triad of prolonged QT interval, U waves, and T-wave inversion.

Arrhythmias are seen frequently in patients after a cerebrovascular stroke and are more common in patients with a co-existing cardiac disease. Other factors that increase the probability of development of arrhythmias in these patients include diabetes mellitus, hypertension, and increasing age. An independent predictor tool for the development of arrhythmias is the NIHSS score. The most common arrhythmias seen in patients with acute stroke are atrial fibrillations, followed by sinus tachycardia, premature ventricular complexes, and ventricular tachycardia.

Two-dimensional (2D) echocardiographic features

Neurogenic stunned myocardium can present with poor left ventricular function. Banki et al. evaluated patients with subarachnoid hemorrhage and cardiac dysfunction and showed that the cardiac wall motion abnormalities in these patients matched the changes seen on their ECGs [15].

Management

The prevalence of asymptomatic coronary artery disease is high in patients of acute ischemic stroke. These two entities have similar risk factors and are, thus, common in the same subset of the population. Considering the coexistence of these conditions, it is essential to assess patients of stroke for cardiovascular abnormalities and dysfunction. Also, due to the impaired cognition and functional capacity of stroke patients, there is a high likelihood of asymptomatic cardiac dysfunction in them. Additionally, cardiac injury and dysfunction is an important cause of morbidity and mortality in such patients. Because of all these factors, cardiac monitoring is especially crucial in these patients with stroke [6].

As per the American Heart Association/American Stroke Association (AHA/ASA), patients with ischemic stroke or transient ischemic attack (TIA) should be subjected to cardiovascular risk assessment, followed by aggressive risk reduction management. The guidelines also recommend that patients with multiple risk factors for coronary heart disease or a high Framingham score should be subjected to noninvasive testing for coronary artery disease. The choice of investigation can also be determined by the ACC/AHA guidelines. Lastly, the management of the patient should be individualized and modified according to the patient’s clinical scenario. However, if the cardiac dysfunction is due to NSM, coronary angiography is not recommended routinely.

## Conclusions

Against a backdrop of neurological events, cardiac abnormalities can lead to poor outcomes. The pathophysiology of such cardiac dysfunction lies in the increased release of catecholamines due to neurologic damage, eventually leading to myocardial necrosis. Several independent studies have shown that insular involvement is most likely responsible for the autonomic dysfunction in patients of stroke. The clinical features of NSM are similar to acute coronary syndrome, making it difficult to distinguish the two clinically. Moreover, no definite guidelines are currently available concerning the management of NSM. In patients who are at a high risk of developing coronary heart disease, careful risk assessment and aggressive management should be initiated to reduce morbidity and mortality in these patients.
